# A Segmentation Method of Foramen Ovale Based on Multiatlas

**DOI:** 10.1155/2021/5221111

**Published:** 2021-09-20

**Authors:** Jiashi Zhao, Huatao Ge, Wei He, Yanfang Li, Weili Shi, Zhengang Jiang, Yonghui Li, Xingzhi Li

**Affiliations:** ^1^School of Computer Science and Technology, Changchun University of Science and Technology, Changchun 130022, China; ^2^Zhongshan Institute of Changchun University of Science and Technology, Zhongshan 528436, China; ^3^Bethune First Hospital of Jilin University, Changchun 130012, China

## Abstract

Trigeminal neuralgia is a neurological disease. It is often treated by puncturing the trigeminal nerve through the skin and the oval foramen of the skull to selectively destroy the pain nerve. The process of puncture operation is difficult because the morphology of the foramen ovale in the skull base is varied and the surrounding anatomical structure is complex. Computer-aided puncture guidance technology is extremely valuable for the treatment of trigeminal neuralgia. Computer-aided guidance can help doctors determine the puncture target by accurately locating the foramen ovale in the skull base. Foramen ovale segmentation is a prerequisite for locating but is a tedious and error-prone task if done manually. In this paper, we present an image segmentation solution based on the multiatlas method that automatically segments the foramen ovale. We developed a data set of 30 CT scans containing 20 foramen ovale atlas and 10 CT scans for testing. Our approach can perform foramen ovale segmentation in puncture operation scenarios based solely on limited data. We propose to utilize this method as an enabler in clinical work.

## 1. Introduction

Trigeminal neuralgia is a neurological disease that occurs mostly in one or more branches of the facial unilateral trigeminal nerve. The pain is similar to electric strike or tingling-like and is asymptomatic in intermittent periods. It is mainly primary trigeminal neuralgia. In a few cases, trigeminal neuralgia can be secondary to brain tumors or vascular abnormalities [1]. An epidemiological survey study in the United States showed that the incidence of trigeminal neuralgia in men is 2.5 per 100,000, and the incidence in women is 5.7 per 100,000 [2]. The peak prevalence is between 50 and 60 years old, and the prevalence rate increases with age. Among people over 80, the incidence rate is 25.9/100,000 per year [3]. Under normal circumstances, speaking, chewing, brushing teeth, shaving, or even a cool breeze may cause short-term attacks in some patients. The disease causes great trouble to the patients' daily life and easily causes anxiety and depression emotions, even suicide [4].

Clinically, the treatment of trigeminal neuralgia is mainly based on doctors' experience knowledge for puncture and computer-assisted puncture based on radiological information. During the puncture process, the puncture needle needs to pass through the skin and enter the semilunar ganglia from the foramen ovale of the skull. However, the narrow foramen ovale of the skull base in different patients and their different shapes pose great challenges to the surgical process. The key to this operation is to accurately locate the foramen ovale position during the operation [5, 6]. The position of the foramen ovale in the skull base is shown in the red area in Figure 1. Puncture based on empirical knowledge has a high failure rate and a high demand on doctors. Computer-assisted puncture needs to determine the specific location of the foramen ovale before surgery [7]. It takes a long time to manually mark the location and relies on the doctor's personal experience, which is highly subjective. Therefore, precise and rapid segmentation of the foramen ovale at the skull base can effectively improve the success rate of puncture, reduce the length of operation, and relieve the pain of patients.

Medical image segmentation methods widely used domestically and internationally are mainly divided into traditional methods and methods based on deep learning. In traditional methods, the threshold method, region growth method, and map segmentation method are mostly used. The threshold method and the region growing method are simple to implement, but the threshold method is very sensitive to noise and uneven grayscale. The region growing method needs to manually provide a seed point. This method is also very sensitive to noise and may produce discontinuous regions. The two methods are to segment the whole, while our target area is a part of the whole skull. The most popular segmentation method is to use deep learning for segmentation, but deep learning requires a lot of data sets [8], which can explain poorly. In recent years, the atlas segmentation method has gradually become one of the effective methods in the field of medical image segmentation [9]. The work of many scholars has shown that prior knowledge of anatomy can help segment brain images with complex structures, low target area boundary contrast, and large intersubject and intrasubject variance. The atlas-based segmentation method utilizes the most anatomical prior knowledge. In the process of registration, the method minimizes or eliminates the influence of various kinds of noise on the segmentation results and has good robustness. Asim et al. [10] use a multiatlas method to divide the brain according to different atlases and then combine the features extracted from these anatomical units to comprehensively and accurately detect Alzheimer's disease. Bao et al. [11] proposed a multimode and multiatlas feature representation method and used a two-step feature selection method to select the most characteristic features for the classification of schizophrenia. Tor-Díez et al. [12] used a multiatlas segmentation method for the analysis of children's brain structure. The cortex is the region of interest for this problem. They proposed a block-based nonlocal model and iterative optimization scheme, which can provide reliable cortical segmentation. As a result, it is of great significance in predicting children's developmental health information. Su et al. [13] proposed a multiatlas segmentation method optimized for the thalamus, which can accurately quantify the thalamus and volume and can track the development of some neurological diseases in time. Boucher et al. [14] realized the automatic segmentation of the lateral ventricle by using a deformable multiatlas segmentation algorithm for ultrasound and MRI fusion using local linear correlation metrics, which can be used to evaluate the brain development of newborns. van der Heyden et al. [15] used a multiatlas method to automatically segment the healthy tissue around the tumor during radiotherapy, which improved the current situation of clinical doctors manually describing the healthy tissue. Tang et al. [16] introduced the multiatlas segmentation method to the segmentation of brain tumor images and adopted a new low-rank method that uses spatial constraints to obtain restored images containing normal brain regions.

This article comprehensively determines the effectiveness of the multiatlas segmentation technology for the segmentation of the skull base foramen ovale and proposes a segmentation method for skull base foramen ovale based on multiatlas. Through a large number of investigations and studies, we find that we apply the multiatlas segmentation method to the segmentation of the foramen ovale in the skull base for the first time and created the foramen ovale atlas data set of the skull base for the first time. This method selects the 10 atlas images that are most similar to the image to be segmented from the atlas set according to the normalized cross-correlation similarity measure, and then, the method based on multiresolution affine transformation and multiresolution B-spline transformation is used to perform coarse registration and fine registration on the image to be segmented and the image selected from the atlas. Finally, the STAPLE [17] algorithm is used to fuse the label images to obtain the final predicted segmentation results. We also compared the segmentation effects of the MV [18] algorithm and the SIMPLE [19] algorithm. The results show that the segmentation method based on atlas can be applied to the segmentation of the foramen ovale at the base of the skull. We have completed the segmentation of the foramen ovale at the base of the skull under low data conditions, with high accuracy to meet the needs of clinical surgery.

## 2. Materials and Methods

The multiatlas segmentation method has gradually become one of the commonly used methods in the field of medical image segmentation. This method has three steps: image similarity selection, multiatlas registration, and label fusion.

### 2.1. Atlas Segmentation Method

The atlas consists of two parts: a grey image and its corresponding manually segmented label image. The segmentation method based on the atlas is equivalent to transforming the segmentation problem into a registration problem. In the image registration, the floating image is matched with the fixed image through deformation. The image to be segmented here is used as the fixed image, and the image selected from the atlas for registration with the fixed image is used as the floating image. According to the number of atlases required for registration, atlas segmentation is divided into single atlas segmentation and multiple atlas segmentation. The steps of multiatlas segmentation are mainly divided into three steps. Firstly, we find several moving images that are most similar to the fixed image from the atlas. Secondly, it is indispensable to register the selected moving image with the fixed image to obtain the corresponding transformation matrix *T* and then apply the transformation matrix *T* to the marked image corresponding to the moving image. Finally, label fusion is performed on all the transformed atlas label images to obtain the final segmentation result. The segmentation process is illustrated Figure 2.

Human brain images are more complex, and the use of multiple atlases for registration and fusion largely compensates for the insufficient registration effect that may be caused by the inappropriate selection of a single atlas. However, Aljabar et al. [20] found that the segmentation accuracy does not completely increase with the increase of the number of atlases, and the more the number of atlases, the time for segmentation calculation will also increase linearly. Awate et al.'s research [21] shows that the most appropriate number of atlases is about 10. Therefore, this article will select 10 moving images from the atlas for registration with the fixed image.

### 2.2. Registration Technology

Registration is a crucial part of the multiatlas segmentation process. The quality of the registration algorithm has a direct impact on the final segmentation result. The registration process in this article is divided into two steps. The first step is to use a registration method based on multiresolution affine transformation to act on the reference image and the floating image for coarse registration, and the second step uses the registration method based on multiresolution B-spline transformation to perform the fine registration on the fixed image and the moving image.

Multiresolution is a strategy often used in medical image registration. It refers to sampling the image to increase or decrease the resolution of the image, so that it is convenient for further processing of the image. Firstly, the medical image is smoothly processed by a low-pass filter to prevent the image from being interfered by noise during the acquisition and transmission process, improves the quality of the medical image, and obtains an image with a constant scale. Then, downsample the fixed image and the moving image. The image can generate several images with different resolutions to form an image pyramid. Hierarchical registration is essentially a coarse-to-fine registration strategy. At the beginning, the optimal parameters are searched for in the low-resolution layer. Although the image information of this layer is not complete and the registration accuracy is not high, the registration parameters obtained are close to the optimal solution, and the amount of image data of this layer is small, which reduces the time required for registration. After multilevel registration, accurate image registration results can be obtained in the last layer, and at the same time, local convergence problems that occur during single-level registration can be avoided. The multiresolution registration flow chart is shown in Figure 3.

The B-spline transformation function achieves the effect of nonrigid registration by moving the control points, which can control local deformation. The specific displacement of the control point is calculated by the optimization algorithm, so as to achieve the effect of simulating any nonlinear transformation. First, the fixed image is gridded, and the points on the image become control points after gridding. We assume that the position of a control point in the two-dimensional image is *φ*_*i*,*j*_ and the grid spacing is *δ*_*x*_ × *δ*_*y*_; based on the consideration of accuracy and efficiency, the uniform third-order B-spline basis function is usually selected for image registration, then the B-spline transformation of any point (*x*, *y*) on the moving image can be expressed as

(1) $$\begin{array}{c} T\left(x,y\right)=\overset{3}{\underset{m=0}{\sum }}\;\overset{3}{\underset{n=0}{\sum }}\;B_{m}\left(u\right)B_{n}\left(v\right)\varphi_{i+m,j+n}. \end{array}$$

In the formula, *φ*_*i*+*m*,*j*+*n*_ represents the coordinate positions of the nearest 4 × 4 control points; the *i* and the *j*, respectively, represent the position index of the adjacent control points, *i* = ⌊*x*/*δ*_*x*_⌋ − 1, *j* = ⌊*y*/*δ*_*y*_⌋ − 1; ⌊⌋ represents the round-down function; *m* and *n* are the order of B-spline basis functions; *u* and *v* are the relative unit control grid positions of (*x*, *y*), *u* = (*x*/*δ*_*x*_) − ⌊*x*/*δ*_*x*_⌋, *v* = (*y*/*δ*_*y*_) − ⌊*y*/*δ*_*y*_⌋; *B*_*m*_(u) represents the *m*-th B-spline basis function; and the expressions are as

(2) $$\begin{array}{c} \left\{\begin{array}{c} B_{0}\left(\text{u}\right)=\frac{{\left(1-u\right)}^{3}}{6},\\ B_{1}\left(u\right)=\frac{3u^{3}-6u^{2}+4}{6},\\ B_{2}\left(u\right)=\frac{-3u^{3}+3u^{2}+3u+1}{6},\\ B_{3}\left(u\right)=\frac{u^{3}}{6}. \end{array}\right. \end{array}$$

Among them, 0 ≤ *u* < 1, these functions act as weighting functions, and they weight the influence of each control point on *T*(*x*, *y*) according to the distance from the control point to (*x*, *y*).

### 2.3. Label Fusion

This paper uses the STAPLE algorithm to complete the label fusion step. The STAPLE algorithm uses the maximum expectation algorithm iteration to estimate the performance parameters and probability distribution. In the fusion process, it is equivalent to treating each atlas as a weak classifier, using the maximum expectation estimation to set the weight of each classifier and then fusing to obtain the final segmentation result. At the same time, we used the majority voting algorithm (MV) for tag fusion and the SIMPLE method to complete the fusion as a comparison experiment. The MV algorithm is a method to determine the final fusion label value according to the criterion that the minority obeys the majority. The SIMPLE method combines atlas selection and evaluation strategies and gradually reduces the number of maps through selective iteration to achieve a good fusion effect.

## 3. Results and Discussion

### 3.1. Construction of Data

In this paper, on the human skull CT, the foramen ovale on the left and right sides of the skull base are segmented separately. The experimental data comes from the Second Hospital of Jilin University, and the inclusion criteria are (1) a complete whole skull and (2) people who are 20 years old and above. A total of 30 CT data are obtained by screening according to the above criteria. Then, under the guidance of professional physicians, 20 data are selected to make the atlas, and the remaining 10 data are used for experimental testing. (Note: all data were obtained with the patient's knowledge and consent.) The preparation steps of the atlas are as follows: firstly, the threshold method and the region growing method are applied to process the CT data. Secondly, the foramen ovale area at the base of the skull was manually segmented. Finally, a slight Gaussian smoothing on the data is performed. A set of atlases contains atlas images and their corresponding label images. One of the sets of the atlas made is shown in Figure 4.

### 3.2. Experiment and Parameter Setting

In the entire experimental process, firstly, the 10 images with the highest similarity to the fixed image are selected in the atlas using the normalized cross-correlation similarity measurement method for registration. The normalized cross-correlation formula is defined as follows:

(3) $$\begin{array}{c} \text{NCC}\left(\tau ,\text{TI},\text{FI}\right)=\frac{\sum_{i=1}^{n}\left(\text{TI}\left(x_{i}\right)-\bar{\text{TI}}\right)\times \sum_{i=1}^{n}\;\left(\text{FI}\left(\tau \left(x_{i}\right)\right)-\bar{\text{FI}\left(\tau \right)}\right)}{\sqrt{\sum_{i=1}^{n}\;{\left(\text{TI}\left(x_{i}\right)-\bar{\text{TI}}\right)}^{2}\times \sum_{i=1}^{n}\;{\left(\text{FI}\left(\tau \left(x_{i}\right)\right)-\bar{\text{FI}\left(\tau \right)}\right)}^{2}}}, \end{array}$$

(4) $$\begin{array}{c} \bar{\text{TI}}=\overset{n}{\underset{i=1}{\sum }}\frac{TI\left(x_{i}\right)}{n}, \end{array}$$

(5) $$\begin{array}{c} \bar{\text{FI}\left(\tau \right)}=\overset{n}{\underset{i=1}{\sum }}\frac{\text{FI}\left(\tau \left(x_{i}\right)\right)}{n}, \end{array}$$

where  TI(*x*_*i*_)/*n* represents the gray value of pixel *x*_*i*_ in the fixed image,  FI(*x*_*i*_)/*n* represents the gray value of pixel *x*_*i*_ in the moving image, and *n* represents the number of image pixels; considering that CT data may come from different imaging equipment, there are nonstandard intensities between images, so it is selected as the atlas selection criterion.

In the registration process, we use the Elastix [22] toolkit to perform registration based on affine transformation and B-spline transformation. In the above two registration processes, a multiresolution strategy is used. The image is first smoothed by Gaussian kernel filtering, and then, downsampling by a factor of 2 is used for each resolution layer. Considering the generation effect and speed, the interpolation method adopts the linear interpolation method, and the interpolation method used to generate the final segmentation result adopts the third-order B-spline interpolation method. During each iteration, a random sampling method is used to randomly select 2000 voxels to calculate the normalized mutual information value between the images, which improves the speed of the registration optimization parameters, and uses the gradient descent optimization algorithm to optimize the normalized mutual information value. For affine transformation registration, each layer is set to 1000 iterations, which is set to 4 layers. For B-spline registration, each layer is set to 3000 iterations, and a grid spacing of 5 mm is used, which is set to 5 layers.

In the label fusion process, the STAPLE algorithm is used to fuse a single prediction result to obtain the final segmentation result. Here, we also use the MV algorithm and the SIMPLE algorithm for comparison experiments.

### 3.3. Evaluation Index

After obtaining the segmentation results, it is necessary to adopt appropriate evaluation indicators to evaluate the segmentation results of different methods. This paper uses Dice coefficient, 95% Hausdorff distance, and average surface distance (ASD) to verify the accuracy of the segmentation results. The Dice coefficient is used to measure the relative volume overlap between the algorithm segmentation results and the manual segmentation results, and the latter two evaluation standards are used to measure the consistency between the segmentation boundaries. The higher the Dice coefficient, the better the segmentation result. The smaller the Hausdorff distance and the average surface distance, the better the segmentation result. Its definition is as Equations (6), 7, 8, 9, and 10:

(6) $$\begin{array}{c} \text{Dice}\left(A,B\right)=\frac{2V\left(A\cap B\right)}{V\left(A\right)+V\left(B\right)}, \end{array}$$

where *V*(*A*) and *V*(*B*) represent the predicted segmentation result and the volume of the doctor's manual segmentation result, respectively. *V*(*A*∩*B*) represents the volume of the above overlapping part.

(7) $$\begin{array}{c} \begin{array}{c} \text{ASD}=\frac{1}{\left|S\left(A\right)\right|+\left|S\left(B\right)\right|}\left(\underset{a\in S\left(A\right)}{\sum }\;\min_{b\in S\left(B\right)}||a-b||+\underset{b\in S\left(B\right)}{\sum }\;\min_{a\in S\left(A\right)}||b-a||\right), \end{array} \end{array}$$

where *S*(*A*) represents the set of surface voxels of the predicted segmentation result, *S*(*B*) represents the set of surface voxels of the doctor's manual segmentation result. *a* and *b*, respectively, represent a voxel subset of the two voxel sets.

(8) $$\begin{array}{c} H\left(A,B\right)=\max\left(h\left(A,B\right),h\left(B,A\right)\right), \end{array}$$

(9) $$\begin{array}{c} h\left(A,B\right)=\max_{a\in A}\;\left\{\min_{b\in B}||a-b||\right\}, \end{array}$$

(10) $$\begin{array}{c} h\left(B,A\right)=\max_{b\in B}\;\left\{\min_{a\in A}||b-a||\right\}, \end{array}$$

where ‖·‖ represents the Euclidean distance between the two points *a* and *b*.

Testing on 10 data, we use the MV, STAPLE, and SIMPLE methods to perform experiments on the left and right foramen ovale at the base of the skull and then display the average of average Dice, 95% Hausdorff and average surface distance obtained by different methods on the three-line graph obtained by different methods on an average three-line graph. In order to visually show the difference of the segmentation effect obtained by different methods, we also draw box plots of the three methods on each evaluation index.

### 3.4. Experimental Results

Segmentation results of the foramen ovale at the skull base and manual segmentation results are shown in Figure 5. The experimental results show that the three methods can be used to segment the foramen ovale.

The comparison chart of each method and manual segmentation is shown in Figure 6. Red is the result of manual segmentation, and green is the segmentation result of different methods. We can see that the segmentation effect of the MV algorithm is not good, the segmented oval foramen has a discontinuity problem, and the segmentation result is incomplete, which is quite different from the manual segmentation result. STAPLE and SIMPLE segmentation results are better.

### 3.5. Data Analysis and Discussion

The average value of Dice which is obtained from 10 groups of data tested by three methods, MV, STAPLE, and SIMPLE, is shown in Table 1. It can be seen from Table 1 that the average Dice of the foramen ovale on the left of the MV algorithm is 0.790, and the average Dice of the foramen ovale on the right is 0.803. The average Dice of the foramen ovale on the left of the STAPLE algorithm is 0.858, and the right is 0.870. The average Dice of the foramen ovale on the left of the SIMPLE algorithm is 0.853, and the right is 0.871.

The average value of the 95% Hausdorff distance which obtained from 10 groups of data tested by the above three methods is shown in Table 2. From Table 2, it can be indicated that the average 95% Hausdorff distance of the left oval foramen of the MV algorithm is 5.054, and the right is 3.639. The average 95% Hausdorff distance of the left oval foramen of the STAPLE algorithm is 4.274, and the right is 3.452. The average 95% Hausdorff distance of the foramen ovale on the left of the SIMPLE method is 4.644, and right is 3.227.

The average value of ASD which obtained from 10 groups of data tested by the above three methods is shown in Table 3. From Table 3, it can be demonstrable that the average ASD value of the foramen ovale on the left side of the MV algorithm is 1.258, and the average ASD value of the foramen ovale on the right side of the MV algorithm is 0.933. The average ASD value of the foramen ovale on the left side of the STAPLE algorithm is 0.998, and the right is 0.739. The average ASD value of the foramen ovale on the left side of the SIMPLE algorithm is 1.067, and the right side is 0.728. From the data in Tables 1–3, it can be seen that the Dice of MV algorithm segmentation is lower, and the 95% Hausdorff distance and the ASD are higher, indicating that the MV algorithm segmentation effect is poor. The Dice of the STAPLE and SIMPLE algorithms is higher, and the 95% Hausdorff distance and the ASD are lower, indicating that the STAPLE and SIMPLE algorithms have better segmentation effects.

Figures 7–9 sequentially show the left and right foramen ovale Dice box plots, 95% Hausdorff distance box plots, and ASD box plots drawn by the three methods of MV, STAPLE, and SIMPLE for 10 sets of test data. The maximum value, upper quartile, median, lower quartile, and minimum value are displayed on the box plots, which can reflect the overall characteristics of multiple sets of data. The horizontal line in the box plot represents the median number. From the box plots, we can see that the effect of the MV algorithm is relatively poor. The Dice value of the STAPLE algorithm and the SIMPLE method is above the chart, indicating that a better segmentation effect can be achieved for the test image. The median of 95% Hausdorff distance and ASD of STAPLE and SIMPLE methods is below the chart, which also shows that these two methods can achieve better segmentation results for the test image.

## 4. Data Analysis and Discussion

From the above chart data, it can be seen that the segmentation results of the STAPLE method and the SIMPLE method are relatively close, and both are significantly better than MV. This is because the MV method compares and selects the pixel values at the same position of each floating image and chooses the pixel value with the most occurrences as the actual pixels of the position; although the prior information of each floating image is fully considered, all image information is treated equally without considering the difference between each floating image and the fixed image. The SIMPLE method and the STAPLE method consider the difference information between the fixed image and each floating image. The STAPLE method uses the expectation maximization algorithm to calculate the weight coefficient of the floating image, and finally, the weighted average is performed to obtain the final segmentation result. The SIMPLE method assigns weights based on the floating images and the performance level of the fusion result obtained after each iteration are, and in the process of estimating the performance level, floating images with poor performance levels are discarded. Theoretically speaking, the SIMPLE algorithm is better than the STAPLE algorithm [19], because the SIMPLE algorithm discards floating images that do not perform well, but in fact, these floating images may also contain useful information. From the overall experimental results, the segmentation effect of the right foramen ovale is better than that of the left foramen ovale. We think that it may be related to the difference in the structure of the foramen ovale on the left and right sides. But we have consulted relevant academic data, and according to the data, the conclusion is that there is no statistical difference in the length, width, and area of the foramen ovale on both sides [23, 24]. There is currently no exact theory to explain this experimental result.

## 5. Conclusions

Trigeminal neuralgia seriously affects the normal life of patients. In clinical practice, surgical needles are often used to puncture the inside of the foramen ovale at the skull base for radiofrequency ablation. When puncturing the target point, it relies too much on the doctor's personal experience, and the operation is difficult. Computer-assisted puncture based on radiological information can improve the success rate of puncture operations. With the aid of a computer, the doctor performs a puncture based on the information of the foramen ovale region segmented out before the operation and then can accurately reach the target point. During the puncture process, the imaging equipment displays the position of the puncture needle in real time for the doctor to make judgments. Computer-assisted trigeminal neuralgia puncture surgery reduces the pain suffered by patients and the probability of postoperative complications, lowers the threshold of puncture surgery, and improves the success rate of puncture surgery. The current problem is that the preoperative segmentation takes a long time; the average time is about 30 minutes, but it does not affect the real-time puncture work of the assistant intraoperative doctors. The future work is mainly in two aspects. On the one hand, we optimize our segmentation algorithm to reduce the time required during the registration and fusion process, and on the other hand, we improve the segmentation accuracy.

From what has been discussed above, in this paper, a segmentation method for the foramen ovale based on multiatlas is proposed, which provides an idea for foramen ovale segmentation, and can provide great convenience for computer-assisted puncture surgery. This article also creates the skull base foramen ovale atlas data set for the first time, which provides data support for future research on the skull base foramen ovale. The experimental results show that the segmentation of the foramen ovale by the multiatlas method has high accuracy and good effect, and it is expected to be applied in clinical puncture surgery.

## Figures and Tables

**Figure 1:** Bottom view of the skull base.

**Figure 2:** Schematic diagram of multiatlas segmentation method.

**Figure 3:** Schematic diagram of multiresolution registration.

**Figure 4:** A set of the atlas manually segmented.

**Figure 5:** Manual segmentation and the results of segmentation of the foramen ovale structure of the skull base by various algorithms. (a) Segmentation result on the left. (b) Segmentation result on the right. Number 1 is manually segmented images, number 2 is MV algorithm segmentation image, number 3 is STAPLE algorithm segmentation image, and number 4 is SIMPLE algorithm segmentation image.

**Figure 6:** Comparison of the results of each method and manual segmentation. (a) Comparison between segmentation method and manual segmentation on the left. (b) Comparison between segmentation method and manual segmentation on the right. Number 1 is a comparison between MV algorithm and manual segmentation, number 2 is a comparison between STAPLE algorithm and manual segmentation, and number 3 is a comparison between SIMPLE algorithm and manual segmentation.

**Figure 7:** Dice box plots of the foramen ovale on the left and right sides of each method: (a) foramen ovale box plot on the left; (b) foramen ovale box plot on the right.

**Figure 8:** Box plot of the 95% Hausdorff distance of the foramen ovale on the left and right sides of each method: (a) foramen ovale box plot on the left; (b) foramen ovale box plot on the right.

**Figure 9:** Box plot of the average surface distance of the foramen ovale on the left and right sides of each calculation method: (a) foramen ovale box plot on the left; (b) foramen ovale box plot on the right.

**Table 1:** Dice average of segmentation results of different methods.

Dice	Left foramen ovale	Right foramen ovale
MV	0.790	0.803
STAPLE	0.858	0.870
SIMPLE	0.853	0.871

**Table 2:** The average value of 95%Hausdorff distance of the segmentation results of different methods.

95%Hausdorff distance	Left foramen ovale	Right foramen ovale
MV	5.054	3.639
STAPLE	4.274	3.452
SIMPLE	4.644	3.227

**Table 3:** Average surface distance average of segmentation results of different methods.

ASD	Left foramen ovale	Right foramen ovale
MV	1.258	0.933
STAPLE	0.998	0.739
SIMPLE	1.067	0.728

## Data Availability

The data used to support the findings of this study are available from the corresponding author upon request.
